The article "Effects of Autophagy-Related Genes on the Prognosis and Immune Microenvironment of Ovarian Cancer" was published in 2022. Journal: Biomed Res Int.

# Effects of Autophagy-Related Genes on the Prognosis and Immune Microenvironment of Ovarian Cancer

**DOI:** 10.1155/2022/6609195

**Published:** 2022-07-30

**Authors:** Jing Zhang, He Yan, Yan Fu

**Affiliations:** ^1^Department of Obstetrics and Gynecology, The First Hospital of Jilin University, Xin Min Street 71, 130021 Changchun, China; ^2^Department of Emergency Medicine, The First Hospital of Jilin University, Xin Min Street 71, 130021 Changchun, China

## Abstract

Ovarian cancer (OC) is among the most malignant tumors of the female reproductive system. The role of autophagy in cancer is complex, and the functional relationship between autophagy-related genes and OC remains unclear. Here, the prognostic value of autophagy-related genes in OC and relationships between autophagy and immune function were evaluated. OC data from The Cancer Genome Atlas and the Human Autophagy Database were obtained to identify autophagy-related genes. Univariate and multivariate Cox analyses were used to construct a prognostic model based on autophagy-related genes. Relationships between risk scores and clinical traits were evaluated. Gene Ontology (GO), Kyoto Encyclopedia of Genes and Genomes (KEGG), and Cytoscape were used to analyze gene functions and their effects on the immune microenvironment. Relationships between autophagy genes and long noncoding RNAs (lncRNAs) were evaluated by Pearson's correlation coefficients, and lncRNAs corresponding to the autophagy-related genes associated with OC prognosis were used to construct a model. Relationships between risk scores and survival and prognosis were evaluated. Finally, a gene set enrichment analysis was performed. Seven autophagy-related genes (CAPN1, CDKN1B, DNAJB1, GNAI3, MTMR14, RHEB, and SIRT2) were identified as independent predictors of prognosis. Three lncRNAs corresponding to autophagy genes independently influenced prognosis. Autophagy genes are closely related to immunity. Fifteen immune cell types showed different levels of infiltration between the high- and low-risk groups. Moreover, immune cell infiltration differed between the high- and low-risk groups based on the model. Our analysis of genes and lncRNAs related to prognosis clarifies the role of autophagy in OC and provides a theoretical basis for further research.

## 1. Introduction

Ovarian cancer (OC) is the fifth most lethal cancer in women and accounts for more than 150 000 deaths annually worldwide. The mortality rate of OC has increased over the past few years [1, 2]. Despite recent improvements in cytoreductive surgery and chemotherapy, the 5-year survival rate of OC remains approximately 30%–40% owing to late diagnosis and chemoresistance [3, 4].

The article "Effects of Autophagy-Related Genes on the Prognosis and Immune Microenvironment of Ovarian Cancer" was published in 2022. Journal: Biomed Res Int.

Long noncoding RNAs (lncRNAs) are defined as nonprotein-coding RNA transcripts more than 200 nucleotides in length and are classified into five categories on the basis of their locations relative to nearby protein-coding genes: (1) sense lncRNAs, (2) antisense lncRNAs, (3) bidirectional lncRNAs, (4) intronic lncRNAs, and (5) intergenic lncRNAs [5]. lncRNAs are essential for general cell functions and play roles in the proliferation, migration, and invasion of cancers, including OC [6, 7].

Autophagy is a degradation pathway that is highly conserved during the evolution of eukaryotes. The formation of a double-layer membrane structure allows the transportation of damaged organelles, misfolded and aggregated proteins, and other macromolecular substances to the lysosome for degradation or recycling [8]. Autophagy plays very complex roles in tumors, including inhibiting or promoting them in different environments and stages of cancer development [9, 10]. Autophagy is generally beneficial during the normal state of the body and the early stages of tumors, by eliminating oncogenic protein substrates, misfolded proteins, and damaged organelles, maintaining cell homeostasis, and either preventing tumors from occurring or inhibiting their progression [11]. However, once tumor develop to an advanced stage, autophagy—as a dynamic degradation and recycling system—promotes their survival and growth by enhancing the living ability of cancer cells in an environment characterized by nutrient starvation and hypoxia [12, 13]. Numerous studies have found a close link between autophagy and ovarian cancer. However, further research is required to identify the specific autophagy-related genes which are involved. In this investigation, we constructed a model to accurately identify the prognostic risk for ovarian cancer by screening the associated autophagy genes. Through model validation, it was found that this method could be used as an independent factor for the prognosis of ovarian cancer. Earlier studies found that lncRNAs also play an important role in the occurrence and development of ovarian cancer. We thus also studied the effect of autophagy gene-related lncRNAs on prognosis and constructed a lncRNA model. However, the gene model was more accurate than the lncRNA model, as it had a higher prediction accuracy. In addition, we also found that the autophagy gene model was closely related to immunity. In this study, we have explained the prognostic relationship between autophagy and ovarian cancer from the perspective of biological information, to help aiding in the search for new ovarian cancer prognostic markers.

## 2. Materials and Methods

### 2.1. Data Acquisition and Collation

Microarray data and corresponding clinical data were obtained from 380 OC samples from The Cancer Genome Atlas (TCGA). The Human Autophagy Database (http://autophagy.lu/clustering/index. html) was used to identify all genes involved in autophagy. The CytoHubba plug-in of Cytoscape was used to produce and generate a graph showing the correlations between gene expression levels. All mRNA levels were log2-transformed. Pearson's correlation coefficients were calculated for relationships between gene and lncRNA levels. Values of |*R*2| > 0.3 and *P* < 0.05 were considered significant.

The article "Effects of Autophagy-Related Genes on the Prognosis and Immune Microenvironment of Ovarian Cancer" was published in 2022. Journal: Biomed Res Int.

### 2.2. Model Construction

A univariate Cox analysis of the autophagy-related genes was carried out using the survival package in R, and genes with coxPfilter = 0.05 were screened out. Then, the COXPH command in R was used to conduct a multivariate Cox analysis of these genes, and the coefficients (i.e., hazard ratios (HR) values) were obtained. The data of the obtained genes were used to construct a model. The risk for each sample was assessed using a risk score. The higher the risk score, the worse the prognosis for the patient, and in contrast, the lower the risk score, the better the prognosis for the patient. The risk score for each sample was obtained by multiplying the coefficient for each gene in the model and taking the sum of these products. TCGA samples were randomly divided into training and test groups, and the median risk score for each group was set as the boundary to divide samples into high- and low-risk groups (see attachment 1 for details). Univariate and multivariate Cox analyses of lncRNAs were performed following similar methods to those used for gene-based analyses.

### 2.3. Receiver Operating Characteristics (ROC)

The survivalROC package in R was used to analyze the accuracy of the model. The accuracies of the gene-based model and the lncRNA-based model were compared.

### 2.4. Gene Set Enrichment Analysis (GSEA)

GSEA was used to study pathway enrichment in the high- and low-risk groups. After importing the data for high- and low-risk groups, the gene set database (c2.cp.kegg.v7.4.symbols.gmt) was used for gene set permutations, with 1000 permutations to evaluate significance. Meaningful channels were selected, and R packages plyr, ggplot2, grid, and gridExtra were used to combine pathway results.

### 2.5. Analysis of Immune Infiltration Using CIBERSORT

CIBERSORT was used to analyze the infiltration of immune cells [14]. Levels of immune cell infiltration in each sample were first calculated using CIBERSORT in R. The infiltration of immune cells was plotted using the limma and ggpubr packages in R.

## 3. Results

### 3.1. Construction of an Autophagy-Related Gene Model for Ovarian Cancer

Autophagy-related genes were sorted according to the degree of correlation between expression and prognosis (Figure 1(a), where darker colors indicate stronger correlations) (see attachment 3 for details). Sixteen genes were closely related to prognosis in OC, as determined by univariate Cox analyses: *ATG9A*, *CAPN1*, *CDKN1B*, *CXCR4*, *DNAJB1*, *EGFR*, *FADD*, *GNAI3*, *IL24*, *MTMR14*, *NPC1*, *PPP1R15A*, *RB1*, *RHEB*, *SAR1A*, and *SIRT2* (Figure 1(b) , *P* ≤ 0.05). A multivariate Cox analysis of the 16 genes revealed that *CAPN1*, *CDKN1B*, *DNAJB1*, *GNAI3*, *MTMR14*, *RHEB*, and *SIRT2* were independent factors affecting prognosis. Using the coefficients from the multivariate analysis, these seven autophagy-related genes were used to construct a prognostic model. The purpose of the univariate and multivariate Cox analysis was to determine which autophagy genes were related to ovarian cancer prognosis. In Figure 1, green indicates that the hazard ratio is <1 (low risk), indicating that the higher the gene expression value, the better the prognosis of the patient will be. Red corresponds to a hazard ratio > 1 (high risk), indicating that a higher gene expression value correlates to a worse prognosis (Figures 1(b) and 1(c)).

The article "Effects of Autophagy-Related Genes on the Prognosis and Immune Microenvironment of Ovarian Cancer" was published in 2022. Journal: Biomed Res Int.

### 3.2. Verification of the Autophagy Model

Using the newly established prognostic model, the risk score for each sample was obtained. There were significant differences between patients with high and low risk scores in the training and test groups (Figures 1(d) and 1(e); *P* < 0.001). The accuracy of the model was verified by an ROC analysis; the area under the curve (AUC) values for both the training and test groups were greater than 0.5 (0.779 and 0.641, respectively), indicating that the model was reliable (Figures 1(f) and 1(g)). The risk scores for each patient in the two groups are shown in Figures 2(a) and 2(b). Survival was longer in the low-risk group than in the high-risk group (Figures 2(c) and 2(d)). Figures 2(e) and 2(f) summarizes gene expression profiles in the high- and low-risk groups. We studied the expression of genes in the high-risk group and relationship between gene expression levels and risk scores. The expression of levels of *CDKN1B*, *GNAI3*, and *Sirt2* differed between the high- and low-risk groups, and *CDKN1B* and *Sirt2* levels were positively correlated with the risk score. *GNAI3* expression was negatively correlated with the risk score (Figure 2(g)).

### 3.3. Relationships between the Autophagy Model and Clinical Parameters

Because OC is relatively rare, a univariate analysis including age, grade, and risk score was conducted. Age and risk score had an effect on prognosis in both groups (Figures 3(a) and 3(b)). A multivariate Cox analysis showed that age and risk score in the training group were independent factors affecting prognosis (Figure 3(c) , *P* < 0.05), whereas age, grade, and risk score in the test group could not be regarded as independent predictors of prognosis (Figure 3(d)). We further generated a nomogram for the prediction of 1-, 2-, and 3-year survival (Figure 3(e)).

The article "Effects of Autophagy-Related Genes on the Prognosis and Immune Microenvironment of Ovarian Cancer" was published in 2022. Journal: Biomed Res Int.

### 3.4. Effect of lncRNAs Associated with Autophagy-Related Genes on OC

Abnormal lncRNA expression plays a crucial role in tumor development and progression [8]. Thus, we identified lncRNAs related to the 16 autophagy-related genes associated with prognosis in OC (Figure 4) (see attachment 5 for details). By a univariate Cox analysis, we identified 14 lncRNAs (i.e., LINC02088, AC008115.3, AC027309.1, AC136601.1, AL357153.1, AC022144.1, OSTM1-AS1, AC008659.1, PKP4-AS1, LINC02574, AL355516.1, LINC02273, AC010240.3, and AC011445.1) with prognostic values for OC (Figures 5(a) , *P* < 0.05). A multivariate Cox analysis of these lncRNAs revealed that AC136601.1, LINC02273, and AC011445.1 could independently predict prognosis (Figure 5(b), Stab. 2). Based on the coefficient for each lncRNA, a risk model was developed. There were significant differences in survival between the groups with high and low risk scores (Figure 5(c), *P* < 0.05). A Sankey diagram was generated for an intuitive representation of the impact of the risk score on prognosis, showing that the mortality rate was significantly higher in the high-risk group than in the low-risk group (Figure 5(d)). To compare the accuracy of the gene-based and lncRNA-based models for risk assessment in OC, we generated ROC curves and found that the AUC values for genes were significantly greater than those for lncRNAs, indicating that the model constructed based on autophagy-related genes could more accurately reflect risk in OC (Figure 5(e)).

### 3.5. Associations between Immunity and Autophagy-Related Genes

Our results support the prognostic value of the autophagy-related gene model of OC; accordingly, we performed functional enrichment analyses of genes in the model. A Gene Ontology (GO) enrichment analysis revealed that the genes in the model were enriched in the cell cycle process, cell cycle, and cell growth (Figure 6(a)) (see attachment 6 for details). A Kyoto Encyclopedia of Genes and Genomes (KEGG) enrichment analysis revealed that the genes were involved in pathways related to prostate cancer, gastric cancer, bladder cancer, and other tumor types as well as various immune processes, such as chronic myeloid leukemia, viral protein interaction with cytokine and cytokine receptors, and leukocyte transtumor (Figure 6(b)). A Cytoscape analysis revealed positive regulation of the macrophage migration inhibitory factor signaling pathway and C-C chemokine receptor activity, CXCL12-activated CXCR4 signaling pathway, and other immune-related processes (Figure 6(c)). A GSEA revealed enrichment for apoptosis, hypoxia, IL-2-STAT5 signaling, IL-6-JAK-STAT3 signaling, and other signaling pathways (Figure 6(d)), all of which are related to immunity.

The article "Effects of Autophagy-Related Genes on the Prognosis and Immune Microenvironment of Ovarian Cancer" was published in 2022. Journal: Biomed Res Int.

### 3.6. Relationship between the Autophagy Model and the Immune Microenvironment

Our functional enrichment analyses suggested that there is a close relationship between the model and immunity; therefore, we studied immune cell infiltration in low- and high-risk groups (Figure 7(a)). Levels of infiltration of B cells, CD8+ T cells, dendritic cells (DCs), interdigitating cells (IDCs), macrophages, mast cells, neutrophils, natural killer (NK) cells, plasmacytoid dendritic cells (PdCs), T helper cells, T follicular helper (Tfh) cells, Th1 cells, Th2 cells, tumor-infiltrating lymphocytes (TILs), and Tregs differed between groups (Figure 7(b)). There were significant differences in antigen presenting cell (APC) costimulation, CCR, checkpoint, cytolytic activity, human leukocyte antigen (HLA), inflammation promotion, inflammation, T cell costimulation, T cell costimulation, and type II IFN response in the immune processes (Figure 7(c)).

## 4. Discussion

Autophagy is a tightly regulated and highly conserved lysosomal degradation pathway [15]. The response of autophagy to homeostasis plays an important role in mammalian development and differentiation [16]. The absence or dysregulation of autophagy is associated with a variety of diseases [17]. We examined the effects of autophagy on OC. We first screened autophagy-related genes related to OC prognosis by a Cox regression analysis to build a predictive model. Some of the genes included in these models are closely related to the occurrence and development of OC based on the previous studies. For example, *CAPN1* is the target of adhesion-associated protein hydrolysis [18]. In OC, BRCA1 affects the migration of tumor cells by regulating *CAPN1* [19] and plays an important role in double-stranded DNA damage repair via its interaction with *SIRT2* [20]. Li and Tang found that low levels of *CDKN1B* are associated with a poor prognosis in epithelial ovarian carcinoma [21]. *GNAI3* is involved in the immune pathway in OC [22]. *DNAJB1* and *RHEB* expressions have also been reported to be affected in OC [23, 24]. However, the role of *MTMR14* in OC has not been reported, and further studies on this gene are needed.

The article "Effects of Autophagy-Related Genes on the Prognosis and Immune Microenvironment of Ovarian Cancer" was published in 2022. Journal: Biomed Res Int.

OC is currently diagnosed by ultrasound combined with serum tumor marker analysis [25]. However, the specificity of this method is low, with a 5-year survival rate of only 30%–40% [26]. Therefore, more effective tumor markers are needed to improve the early detection rate of OC. We observed a significant difference in survival between the high- and low-risk groups based on our newly developed predictive model. Furthermore, the accuracy was verified by an ROC curve analysis (AUC > 0.6), supporting its potential use for the early detection of OC. Combinations of biomarkers can improve detection efficiency over those of single markers [27, 28]. To further study the prognostic value of the model, we included clinical parameters in regression analyses and found that the model is an indicator for predicting prognosis, similar to age; however, in a multivariate Cox analysis of the test group, age, grade, and model were not statistically significant. This may be related to the small sample size. Most patients in the sample were classified as grade 2 or 3, whereas only a few patients were classified as grade 1 or 4, making it difficult to accurately evaluate the impact of grade on prognosis. Based on the model, we drew a nomogram, providing a tool for the individualized evaluation of prognosis.

lncRNAs play important roles in all stages of gene expression [29]. A previous study has confirmed that lncRNAs can be used as prognostic biomarkers for OC [30]. Therefore, we screened lncRNAs related to autophagy-related genes and identified lncRNAs related to OC prognosis by univariate and multivariate analyses. In addition to AC011445.1, the three lncRNAs used for modeling have been associated with OC [31], and the other two have not yet been reported in OC. Using the model based on lncRNAs, there were significant differences in prognosis between the high- and low-risk groups. These results indicate that the lncRNA-based model can be used as a biomarker to predict the prognosis in OC. We compared models constructed based on autophagy-related genes and lncRNAs and found that the accuracy of the gene-based model was higher. This comparison is helpful for the selection of effective tumor markers for the early diagnosis of OC in the future.

To gain a deeper understanding of the model constructed by autophagy-related genes, we performed pathway enrichment analyses. The P53 and PI3K-Akt-mTOR pathways play important roles in the activation and regulation of autophagy [32, 33]. Other pathways, involving inflammatory cells, IL2-STAT5, and IL-6-JAK-STAT3, are mainly associated with inflammation and immunity. In fact, OC cells release cytokines to recruit activated stromal fibroblasts and immune cells, leading to inflammatory infiltration in the stroma. This, in turn, impedes the immune response and promotes the proliferation of tumor cells. Wang et al. found that several products of OC inhibit the expression of IL-2R*β*, *γ*, and JAK3, as well as the phosphorylation of STAT5 tyrosine in T cells, thereby inducing immunosuppression in OC [34]. In our study, we also found obvious differences in the activation of cytolytic and inflammation-promoting functions between the high- and low-risk groups. A large number of studies have shown that autophagy is a key regulator of the natural immunity in tumor cells [35]. For example, autophagy can affect IL-1-dependent secretory processes via IL-17, IFN-*γ*, and IL-22 signaling [36]. Autophagy can also regulate T and B lymphocytes and plays an important role in the activation, metabolism, and proliferation of T cells [32, 37]. This is consistent with our results, indicating significant differences in the infiltration of B cells and multiple T cell subsets between the high- and low-risk groups. Autophagy is also closely related to apoptosis and hypoxia. The relationship between autophagy and apoptosis is subtle. During chemotherapy, autophagy can protect tumor cells from apoptosis and eventually result in drug resistance [38]. Excessive autophagy can also lead to apoptosis. In the process of hypoxia, tumor cells use autophagy to undergo metabolic reprogramming to obtain the energy needed for survival [38].

The article "Effects of Autophagy-Related Genes on the Prognosis and Immune Microenvironment of Ovarian Cancer" was published in 2022. Journal: Biomed Res Int.

## 5. Conclusions

In our study, we evaluated the effect of autophagy on prognosis in OC and explored the functions of autophagy. These findings provide direction for the identification of additional tumor markers, including lncRNAs related to the prognosis, and for analyses of the mechanisms underlying the effect of autophagy on OC. A limitation of this study is that the sample size was small and data were obtained from a single database; therefore, a larger sample size and more data are needed to verify the prognostic value of our model. In addition, our results need to be confirmed in large-scale clinical trials. These follow-up studies are expected in the near future.

## Figures and Tables

**Figure 1:** Predictive model for ovarian cancer prognosis based on autophagy-related genes. (a) Relationships between expression levels of autophagy-related genes. Darker colors indicate a stronger relationship. (b) Prognostic autophagy-related genes were screened by a univariate Cox analysis. (c) Establishment of an autophagy risk model by a multivariate Cox analysis. (d and e) Spearman's correlation analysis of relationships between seven autophagy genes in the training and test sets. (f and g) ROC curves showing the predictive efficacy of the autophagy risk signature in training and test sets. ROC: receiver operating characteristics.

The article "Effects of Autophagy-Related Genes on the Prognosis and Immune Microenvironment of Ovarian Cancer" was published in 2022. Journal: Biomed Res Int.

**Figure 2:** Distribution of risk scores in patients with ovarian cancer. (a and b) Distribution of risk scores in the high and low autophagy groups in training and test sets. The *x*-axis indicates the patient number, and *y*-axis indicates the risk score. (c and d) Distribution of survival in the high and low autophagy groups in training and test sets. Dots represent patient status ranked by the increasing risk score. The *x*-axis shows the patient number, and *y*-axis shows the survival time. (e and f) Heatmap showing expression levels of seven genes used to construct the autophagy model in the high- and low-risk groups from training and test sets. (g) Expression of seven genes included in the autophagy model in the high- and low-risk groups; relationships between the expression levels of seven genes and risk scores.

**Figure 3:** Prognostic value of the autophagy risk signature in ovarian cancer. (a and b) Univariate Cox analysis of the effects of age, grade, and risk score on prognosis in ovarian cancer in the training and test groups. (c and d) Multivariate Cox analysis of age, grade, and risk score for the identification of independent risk factors for ovarian cancer in the training and test groups. (e) Nomogram showing the predictive value of the autophagy model for survival at 1, 2, and 3 years.

**Figure 4:** Autophagy genes related to ovarian cancer prognosis (shown in yellow) and corresponding lncRNAs (shown in blue). lncRNAs: long noncoding RNAs.

**Figure 5:** (a) Comparison of autophagy-related lncRNA models with gene models. Univariate Cox analysis of autophagy-related lncRNAs related to prognosis (*P* < 0.05). (b) Multivariate Cox analysis was used to screen autophagy-related lncRNAs for model establishment. (c) Survival of patients with high and low risk scores in TCGA. (d) Sankey map to demonstrate the impact of genes and lncRNAs on patient survival. (e) Accuracies of the autophagy gene-based model and the lncRNA-based model for risk assessment were compared by ROC curves. lncRNAs: long noncoding RNAs; TCGA: The Cancer Genome Atlas; ROC: receiver operating characteristics.

**Figure 6:** Functional enrichment analysis of autophagy genes included in the predictive model. (a) GO enrichment analysis of the autophagy model. (b) KEGG enrichment analysis of the autophagy model. (c) Cytoscape analysis of pathways related to genes in the model. (d) GSEA of pathway enrichment. GO: Gene Ontology; KEGG: Kyoto Encyclopedia of Genes and Genomes; GSEA: gene set enrichment analysis.

The article "Effects of Autophagy-Related Genes on the Prognosis and Immune Microenvironment of Ovarian Cancer" was published in 2022. Journal: Biomed Res Int.

**Figure 7:** Effects of autophagy model on the immune microenvironment. (a) Immune cell infiltration in the high- and low-risk groups based on the predictive model. (b) Box plots of the infiltration of immune cells in the high- and low-risk groups. (c) Box plots of immune function in the high- and low-risk groups.

## Data Availability

The data supporting the findings of this study are available in the Cancer Genome Atlas (TCGA) and the Human Autophagy Database (http://autophagy.lu/clustering/index.html).
